# Refining kill-trap networks for the control of small mammalian predators in invaded ecosystems

**DOI:** 10.1371/journal.pone.0238732

**Published:** 2020-09-08

**Authors:** Andrew M. Gormley, Bruce Warburton

**Affiliations:** Landcare Research–Manaaki Whenua, Lincoln, New Zealand; Texas State University, UNITED STATES

## Abstract

Population control of invasive mammal pests is an ongoing process in many conservation projects. In New Zealand, introduced wild domestic cats and mustelids have a severe impact on biodiversity, and methods to reduce and maintain predator populations to low levels have been developed involving poisoning and trapping. Such conservation efforts often run on limited funds, so ways to minimize costs while not compromising their effectiveness are constantly being sought. Here we report on a case example in a 150 km^2^ area in the North Island, New Zealand, where high predator numbers were reduced by 70-80% in an initial ‘knockdown’ trapping program, using the full set of traps available in the fixed network and frequent checks, and then maintained at low density using maintenance trapping with less frequent checking. We developed and applied a simulation model of predator captures, based on trapping data, to investigate the effect on control efficacy of varying numbers of trap sites and numbers of traps per site. Included in the simulations were captures of other, non-target, introduced mammals. Simulations indicated that there are potentially significant savings to be made, at least in the maintenance phase of a long-term predator control programme, by first reducing the number of traps in large-scale networks without dramatically reducing efficacy, and then, possibly, re-locating traps according to spatial heterogeneity in observed captures of the target species.

## Introduction

Invasive mammalian pests continue to have significant negative impacts on biodiversity values internationally [1–3]. Although some invasive mammals have been successfully eradicated from islands [4, 5], eradication is often not an option on large mainland areas (>100 km^2^), especially where the broadcast application of toxic baits for pest control is socially or politically unacceptable [6]. In such cases the alternative strategic choice is often sustained ‘maintenance‘ control, which attempts to reduce and then hold populations of pests below a threshold density at which their impacts are either eliminated or at least reduced to a level deemed acceptable by stakeholders [7, 8]. In New Zealand, several introduced mammal pests exert a range of negative impacts on conservation and production values [9], among which is a suite of small (<5 kg) predators comprising mustelids and feral cats [10]. These predators are currently managed variably by national and regional government agencies and private conservation initiatives, either singly or as multiple species, using a range of strategic population reduction approaches involving trapping, poisoning, or both [11, 12].

Where landscapes are accessible, fixed networks of kill-traps have the potential to provide long-term maintenance control of mammalian pests in New Zealand [13, 14]. Such approaches can, however, incur high costs due to labour costs associated with trap checking and re-baiting, and maintenance costs associated with trap servicing and replacement [15]. Recent advances have been investigated to reduce these costs, including the implementation of wireless technology to monitor traps remotely for target pest captures, non-target captures, sprung-but-empty traps or bait removal [16]. Given, however, that pest control programmes invariably operate on tight budgets, an imperative to reduce running costs further is ever present.

One potential improvement to reduce cost is refining the layout of the trap network in relation to changing predator numbers. Typically, in a control programme for mammalian pests, an initial ‘knockdown’ phase, where large numbers of pests are removed, is followed by the ongoing maintenance control phase to keep the diminished population at its reduced level [14]. Fixed trap networks have the real possibility that the high number of traps deployed against the initial high predator population will quickly become surplus to requirements for the ongoing, long-term maintenance of the population at a lower density. Refining the ongoing operation of trapping networks in response to anticipated changes in predator population levels would allow freeing-up of the limited resources typically available for pest-control programmes [17] and enable their re-allocation elsewhere. The cost-effectiveness of this type of approach has been debated in overseas examples of mammalian pest control [18], but it has not yet been implemented or trialed in New Zealand.

Poutiri Ao ō Tāne is a pest control programme run by the Hawke’s Bay Regional Council on the east coast of the North Island of New Zealand. This programme uses an infrastructure of kill-traps that target, in particular, three introduced predators: ferrets (*Mustela furo*), stoats (*M*. *erminea*), and feral cats (*Felis catus*). The fixed trap network was established in 2011 with the aim of reducing predator numbers to minimal-impact levels and then maintaining these numbers while minimizing ongoing costs. For the initial knockdown phase, kill-traps were spaced at 200–300 m intervals to ensure all individual predators would be exposed to at least one trap (home ranges of each species typically exceed 50 ha [10, 19]), as per best-practice recommendations for mustelids and cats [20]. To address the issue of cost-minimisation [18], establishment and maintenance of the network has been streamlined by deliberately setting traps along farm access roads and tracks that enable mechanized travel between trap sites and easy access by foot, thereby minimizing transportation and labour costs. After the anticipated initial period of rapid reduction in predator numbers over the period of late 2011 to 2012 [21], the programme has been continued by a maintenance phase since 2013 to suppress predators to low levels continually, using the same network.

In the present study, we first developed an individual-based spatial model of the diminished predator populations [22] and used this to simulate predator trapping across the Poutiri Ao ō Tāne trap network with the aim of determining if a similar number of predators could have been captured with fewer trap sites. We also examined the effect of having multiple traps at each location on the number of predators captured, with both objectives geared towards identifying the most cost-effective means of maintaining low predator numbers. We also examined if those traps removed could be selected based on their capture histories.

## Methods

### Establishment, operation and maintenance of the trap network

The Poutiri Ao ō Tāne trap network was designed and implemented by the Hawke’s Bay Regional Council across ~150 km^2^ in the Hawke’s Bay region of the east coast of New Zealand’s North Island [21], 45 km north of the city of Napier (39.5^o^S, 176.9^o^E; Fig 1). The terrain comprises predominantly rolling to steep farmland ranging from 400 to 1,100 m elevation. In non-farmed areas the land comprises a mixture of exotic scrub vegetation and some remnant patches of native forests at elevations below ~800 m, giving way to more contiguous forest above this level, interspersed with areas of mountain and tussock grasslands at the highest elevations [23].

**Fig 1:** National (a), local (b) maps of the study area. Maps depict (a) the geographical location of Napier city within New Zealand, with the study region indicated by the red square; (b) the Poutiri Ao ō Tāne trap network, with individual trap sites shown by red dots and patches of forest and shrub land indicated by dark and light green shade respectively.

The trapping network was established in 2011 and has been operational since December of that year, comprising 690 kill-traps (DOC 250 model, http://www.doc.govt.nz/documents/conservation/threats-and-impacts/animal-pests/doc250-predator-trap.pdf) set across 15,000 ha (Fig 1). Traps have remained fixed in place since December 2011, with field staff checking them on a monthly basis to record any kills, then clearing and re-setting the traps. For the 30-month duration of this study (December 2011 to May 2014) approximately 50% of the traps were set using either fresh or dried rabbit meat as bait, with the remainder either set but unbaited (December 2011 to December 2012), or set and lured using a prototype synthetic preparation of rat-odour oil (Good Nature Ltd, Wellington, New Zealand) as an attractant (December 2012 onwards).

### Empirical trapping data

Over the 30-month period between December 2011 and May 2014, monthly data on predator captures were accrued and compiled (Wildlife and Environmental Trapping Advancements Ltd, Napier, New Zealand; http://www.bizdb.co.nz/company/9429035740032/). The data included GPS coordinates of all trap locations, all captures (target and non-target species), and all cases of sprung-but-empty traps. Of primary interest were captures of target predators (ferrets, stoats and feral cats), although incidental captures of other mammalian pests were also examined, including possums (*Trichosurus vulpecula*), rabbits (*Oryctolagus cuniculus*), ship rats (*Rattus rattus*), Norway rats (*R*. *norvegicus*), mice (*Mus musculus*), hedgehogs (*Erinaceus europaeus occidentalis*), and weasels (*M*. *nivalis vulgaris*).

Data gathered between December 2011 and May 2013 were not used in simulation modelling, because this time-frame included the large decline in predator numbers during the initial knockdown phase of the newly implemented control programme [24]. Instead, we focused on 12 months of predator data accrued during the maintenance phase of control, from June 2013 through May 2014. This approach was supported by the lower number of captures of target predators in the 3rd year after initiation of the network compared to the first (Fig 2A). Captures over this latter period were aggregated into monthly totals to reflect the schedule of checking traps every month.

**Fig 2:** Predator (a) and non-target (b) mammals captured monthly; data used for simulations are highlighted in light grey. Note the differing dependent-axis scales.

### Trapping simulation model

We developed an individual-based trapping model [22] to simulate monthly captures of the three species of target predators (ferrets, stoats, and cats), and also five of the non-target species (ship and Norway rats, hedgehogs, rabbits and possums), which provided realistic figures for trap competition and saturation (i.e. traps becoming triggered and therefore being out of action until checked again).

In this framework, we simulated animals distributed randomly across the landscape with no constraints with respect to habitat, topography or elevation. The home range of each animal was assumed to be circular and its size defined by σ, the standard deviation of the bivariate normal distribution, where the radius is given by 2.45σ. The probability of animal (*i*) being caught in an empty trap (*j*) was a function of the distance (*d*) between the home-range centre and the trap, as given by:

$$P_{ij}=g_{0}\;\exp\;\left(\frac{-d_{ij}^{2}}{2\sigma^{2}}\right)$$

where g_0_ was the nightly probability of capture in an empty trap located at the centre of its home range [25]. The probability of capture was calculated for each trap+animal combination. Each night, the capture or not for each animal *j*, was calculated as a random draw from a binomial distribution with probability equal to the cumulative probability of capture, calculated as:

$$P_{j}=1-\prod_{i=1}^{T}\left(1-P_{ij}\right)$$

where *T* is the number of available traps that night. Conditional on capture, the actual trap that caught the animal was a random draw from a multinomial distribution with probability *P*_*ij*_.

The three target species all had similar home range sizes and capture probabilities [26] and, therefore, we modelled them as a generic ‘target predator’ (ferret, stoat or cat) with values of g_0_ = 0.05 and σ = 400 m, corresponding to a 95% home-range of c.300 hectares. We based these values on empirical values reported in published literature and reports [19, 27–30]. We modelled the non-target species using g_0_ = 0.05, and σ = 40 m for rats, hedgehogs and rabbits and σ = 65 m for possums, corresponding to 95% home-ranges of 3 and 8 hectares respectively. For both targets and non-targets, we assumed that g_0_ and σ were constant over the simulation period (i.e. bait attractiveness, capture rate and home range size remained constant).

To compare the relative effectiveness of different trap networks, would ideally need the underlying population size to be known, however the only data available are of the actual captures each month. We therefore used a variant of approximate Bayesian computation (ABC, [31]) to estimate the monthly numbers of potentially trappable animals of both target and non-target species (as distinct groups) over the period June 2013 to May 2014. For each monthly data set we initiated the simulation with 200 target and 1,000 non-target animals distributed randomly across the landscape (i.e. with no constraints on home range centres related to habitat, topography or elevation), and then used the trapping model above to simulate captures of the target and non-target groups of species concurrently over a period of 30 days under the full trapping network. After each iteration we compared the number of simulated captures of target and non-target animals with the actual captures for that month (i.e. those in Fig 2). If the simulated captures exceeded the actual captures, the background population size was decreased and vice versa if the simulated captures were lower than the actual captures. The next iteration was then run with the updated background population size. This process was repeated for 200 iterations, by which stage the background population size was relatively stable between iterations (i.e. <20% variation between successive runs). Background population sizes of the target and non-target species from the last 100 iterations were used for the purpose of comparing different levels of trapping effort for each month. Using this approach to estimate the background population size negated the need to model changes in population size due to immigration and breeding.

### Simulation modelling of different trapping effort scenarios

We simulated captures under five levels of trapping effort relative to the actual trap network: all 690 traps (100%) were operational, or 75%, 50%, 33%, or 25% of traps were operational. We constructed the four sets of reduced trap networks by ordering traps by latitude and longitude and then thinning at the appropriate level (e.g. removing every second trap in the ordered list for the 50% trap network). For each level of trapping effort we also simulated four levels of trap capacity at each trap site, ranging from one trap (the actual regime), to two, three or four traps per trap site.

These combinations of trapping effort and trap capacity resulted in 20 sets of simulations (5 levels of trap effort × 4 levels of trap capacity). For each set, the model was run 500 times for each of 12 one-month periods, with the background population size drawn randomly from the 100 simulated background population sizes for that month (estimated previously). We recorded the number of simulated target and non-target animals captured in each iteration, and the results were summed across iterations and months. For each set of simulations we defined the effectiveness of the trapping effort as the number of simulated captures, expressed as a percentage of the captures achieved under the actual trapping layout (i.e. the full trap array with a single trap at each trap site), for both target and non-target species.

## Results

### Effectiveness of the standard trapping network

Between December 2011 and May 2014, the trap network killed a total of 303 predators (Fig 2). Maximum kills occurred during and after the main summer juvenile growth/weaning period and the autumn dispersal period in each year (December to May). As expected, the predator capture rate in the initial knockdown phase, during the first year after commencement of trapping, declined significantly over successive years: an average of 19.2 predators were trapped per month between December 2011 and May 2012, and the trap rate declined by 54% over the next 12 months (June 2012 to May 2013), and by 66% over the subsequent 12 months (June 2013 to May 2014) relative to the first six months. Predator captures showed notable heterogeneity among individual trap sites: of the 690 traps originally deployed, 71% of traps had not captured any target species in the 30 months from December 2011 until May 2014, 19% captured one target predator, 6.5% captured two, and 3.5% of traps captured from three to five predators.

### Simulated captures of predators and of five non-target species

For predators, reducing the percentage of traps set progressively reduced the proportional simulated catch relative to the full network (Fig 3A). Reducing the percentage of traps to 75% and down to 25% of the original trap numbers reduced the mean proportional catch to an average of 95% to 76% of actual captures, respectively (Fig 3A). In contrast, progressive and more substantial changes in predicted simulated non-target captures–up to a 73% decrease–were observed when the proportion of traps set was decreased (Fig 3B). The percentages of simulated non-target animals caught using 75% down to 25% of the original traps were 78% down to 27%, respectively, of the value for a full trap network (Fig 3B).

**Fig 3:** Simulated captures of predators (a) and non-target mammals (b) as a percentage of animals captured under the current trapping configuration. Data points represent the mean relative captures, over twelve one-month trapping sessions, for a range of trapping configurations, each expressed relative to a standard (100%) value of a single trap set per site with all available traps utilized. Vertical lines indicate the 5% and 95% percentile for each combination of the number of traps at each site (1 to 4) and the percentage of trap sites utilized (all, 75%, 50%, 33%, and 25%).

Increasing trap capacity, from a single trap per site to two, three or four traps, resulted in little change in the predicted percentage of either predators or non-target species captured (Fig 3A and 3B). The small changes that were observed were mostly due to the initial doubling from one to two traps per site, but never exceeded a 2% increase; further increases in trap capacity beyond this initial doubling failed to elevate the percentage of captures beyond an additional 0.5% increase.

## Discussion

Strategies for increasing the cost-effectiveness of mammalian pest-control trapping operations, which often run on very limited budgets, include improving accessibility to real-time trap-site information from the trap network,either through logistical improvements in physical access or by facilitating remote-sensing of trap sites [16], and/or by optimizing the spatial arrangement of the trapping network [15, 32]. In the present study we have applied individual-based spatial simulation modelling in the latter context to determine the effect of changing trap densities on predator captures. This could prove to be a cost-effective approach to optimizing the operation of trapping networks, since testing such parameters empirically would be both expensive and time consuming, and would pose a risk of failure if too many traps were removed. Elsewhere, simulation modelling has been used for optimizing insect detection and control networks [33], but we are unaware of such an approach being used for optimizing vertebrate pest-trapping networks, especially one that incorporates competition for traps from non-target species into the model. Tompkins and Ramsey [34] used a similar individual-based spatial simulation approach for optimizing bait-station delivery of fertility control agents to brushtail possums, but because multiple baits could be easily delivered in each bait station they did not have to incorporate the effect of bait loss (or trap occupancy) due to non-target species in their modelling.

Our simulations suggest that, during the maintenance phase of predator trapping, substantial reductions in the number of traps used could still result in similar numbers of captures to those actually obtained using the full network. Simulation results highlighted that even when 75% of traps were removed from the network, approximately 75% of the actual target predators caught would still probably be captured. If the proportion captured needed to be maintained above 90% of what was actually captured, 25% of traps could conservatively be removed (i.e. resulting in 95% of the target animals captured with the full network), or up to 50% could be removed if a less conservative approach was chosen (i.e. 89% of the target animals captured with the full network).

Importantly, these potentially beneficial reductions in trap density will be dependent on the home range of the predators selected in the simulations: the degree to which a trap network can be reduced while maintaining effectiveness against a suite of three species, as here, will be largely dependent on the target species with the smallest home range [35]. In our modelled environment the three target species were all assigned the same home range size (σ = 400 m), although it is worth noting that if ship rats were to be included in simulations as a fourth target species (σ = 40 m), the network would not be able to have up to 50% of the traps removed without substantially reducing its effectiveness for capturing that species. As an additional caveat to changing trap numbers, alterations in the trapping network would also, inevitably, have an impact on the relative capture of non-target species [12]. In our simulations the effect of trap removal was greater on non-target than on target species, due largely to some of the non-target species having smaller home ranges [10]. Indeed, as the trap network was reduced, the mean distance between traps increased, resulting in the simulated home ranges of some non-target animals no longer overlapping with set traps.

The lack of an effect of increasing the trap capacity at each site, in our simulations, was not surprising [22], and is likely to be due to a combination of the relatively low density of both target and non-target species at the study site [21] with no localized aggregations. Also, the nominal length of time between trap checks (i.e. 1 month) along with low pest densities would not be sufficient for the trap network to become saturated. In our simulations, animals were located randomly across the landscape, but if animals were clustered in areas around traps, or if their distribution was influenced by landscape structure [36], trap saturation would be more likely in those areas, and therefore having multiple traps at a site might become more beneficial [22]. This is of practical relevance because of the advent of multi-kill-traps that have recently come to market (http://goodnature.co.nz, https://nzautotraps.com). Such traps are being deployed in a number of predator-free NZ programme sites across New Zealand because of their perceived effectiveness, however, given the example modelled here and the results reported previously[22], there is likely to be little advantage gained from their use.

Empirical trapping data for the capture of target and non-target species (Fig 2) indicate that numerically more non-target mammals were captured than targets in the study area. This, in itself, suggests that competition for traps between target and non-target species could be a factor limiting captures of target predators, and this competition might be reduced if traps or trap-setting could be modified to exclude non-target species, which would in turn increase the traps available for target species and reduce or eliminate any unacceptable trap-induced injuries caused to non-targets [37].

Of the 690 traps originally deployed, >70% of traps caught no target species in 30 months of trapping, in contrast to 3.5% of traps that captured at least three animals. This spatial heterogeneity of predator–trap encounters is a recognized phenomenon in mammalian pest control operations [38] and should also be taken into account for refining trap network performance. In our case, if the traps in locations that had no captures were removed in preference to those traps that had captured several times, the overall effectiveness of the modified trap network might be greater than that simulated and could represent an additional means by which the costs associated with running a trap network could be reduced. However, the difficulty lies in knowing which traps to remove [32]. It may be possible to use initial data to guide which traps to remove. In detailed examination of the data we found that of the 568 traps that had no predator captures in the first 6 months of the study, only 18% (*n* = 104) had subsequent captures over the remainder of the study. In contrast, of the 87 traps that had a target capture in the first 6 months, 41% (*n* = 36) had subsequent captures. In general, traps that caught a target predator in any given fixed-length period were more likely to catch another predator in a subsequent period of similar length. We did not formally explore the reasons for this heterogeneity, but it is likely that environmental factors play a role, especially habitat and landscape: features of habitat connectivity have been shown elsewhere to influence the heterogeneity of captures of small mammals across a landscape [32, 39]. Most markedly in our study, only 10% of traps that had no captures in any 6-month period had captures in the next 6-month period, compared to 22% of traps that had a capture in the first 6 months also having a capture in the next 6 months. Hence, re-arrangement of trap networks in response to these noted effects of spatial heterogeneity on predator captures could represent an additional approach for refining a trap- network, as has been highlighted elsewhere as a possible means of improving the performance of a trapping programme [40].

Overall, the simulation results here indicate there are potentially significant savings to be made, at least in the maintenance phase of a long-term predator control programme, by first reducing the number of traps in large-scale networks without dramatically reducing efficacy, and then, possibly, re-locating traps according to spatial heterogeneity in observed captures of the target species. At the operational level, the true dollar value of such projected savings can be evaluated using existing bio-economic modelling approaches to assess the costs and benefits to pest-control operations [15]. Feasibly, more cost savings could be made via the uptake of emerging technologies, such as applying wireless remote sensing of traps [16], using self-re-setting traps [40], and employing long-life baits to reduce the frequency of trap checks and bait replacement [41]; the latter is becoming more important, as traps in the Poutiri Ao ō Tāne network began to be checked only once every 3 months after mid-2015 (Wendy Rakete-Stones, Hawke’s Bay [New Zealand] Regional Council, pers. comm., 2018). Further, we have identified here that the full extent to which cost savings can be realized will depend on a fuller knowledge of aspects of the target species’ biology relative to their habitat and to the trapping programme, including knowledge of home range sizes, population density (in turn affecting the rate at which traps fill and the network becomes saturated), and the density and relative trapability of the non-target species at the site. In the case of the Poutiri Ao ō Tāne network in particular, but also in the broader context, the approach developed here provides further support for the use of simulation modelling to refine and optimize predator-trapping practices [42, 43]. We suggest that managers of predator-control programmes could benefit from using a similar approach to maximize the impact of operations with limited funding, where the objective is population control rather than eradication [1, 44].
